# Pancytopenia and atrial fibrillation associated with chronic hepatitis C infection and presumed hepatocellular carcinoma: a case report

**DOI:** 10.1186/1752-1947-2-264

**Published:** 2008-08-11

**Authors:** Christopher Labos, Kaberi Dasgupta

**Affiliations:** 1 Department of Internal Medicine, Montreal General Hospital, Cedar Avenue, Montreal, Quebec, H3G 1A4, Canada; 2 McGill University Health Centre, Pine Avenue West, Montreal, Quebec, H3A 1A1, Canada

## Abstract

**Introduction:**

Pancytopenia secondary to hepatitis viral infection is a rare but noted clinical entity. An acute aplastic crisis usually occurs shortly after viral infection, however, viral serologies are usually negative and the pancytopenia is often fatal if left untreated.

**Case presentation:**

A 66-year-old woman presented to the emergency department with shortness of breath and palpitations. She was found to have pulmonary edema secondary to a newly diagnosed atrial fibrillation and was treated with rate control and anticoagulation. She was found to have an anemia that was reported to be longstanding and that was apparently being investigated by a hematologist, although no diagnosis had yet been achieved. Her blood work also revealed a mild leucopenia and pronounced thrombocytopenia. The patient was admitted to ensure appropriate rate control of her atrial fibrillation and for work-up of her pancytopenia. Review of the bone marrow biopsy performed by the hematologist revealed a normal marrow with no infiltrative process. The results of the patient's blood tests ruled out a hemolytic process. There was also no evidence of infection, toxin ingestion, or recent medication that could be associated with pancytopenia. An abdominal ultrasound was ordered to rule out enlargement of the spleen and a possible consumptive coagulopathy. The spleen was mildly enlarged with a diameter of 13 cm. The liver, however, was mildly cirrhotic and a small solitary liver lesion was seen. A magnetic resonance imaging scan of the liver confirmed a single solitary solid mass and the α-fetal protein level in the serum was elevated. The patient's preliminary viral serologies were positive for hepatitis C. The patient was diagnosed with presumed hepatocellular carcinoma and referred to a hepatic surgeon for evaluation of treatment options.

**Conclusion:**

Hepatitis associated aplastic anemia is an acute condition while milder more chronic presentations, such as this case, likely result from increased portal pressure generated from the resulting cirrhosis, which leads to a relative hypersplenism.

## Introduction

A 66-year-old woman presented to the emergency department of the Montreal General Hospital with a 1-week history of dyspnea and recurrent palpitations. She had immigrated to Canada from Ethiopia 20 years previously. At the time of admission, she had been living with her daughter and was active within the household, participating in housekeeping activities. She was being treated by her family doctor for mild hypertension with an angiotensin-converting enzyme inhibitor. However, during the 24-week period prior to admission, she had been followed as an outpatient by the hematology department for moderate but unexplained normocytic anemia (110 g/l; mean corpuscular volume 89 fl), leucopenia (2.7 × 10^9^/liter), and thrombocytopenia (68 × 10^9^/liter). Bone marrow biopsy had not clarified the etiology of her anemia, revealing a normocellular marrow with a slight left shift in the erythroid and myeloid cell lines.

## Case presentation

In the emergency department, an electrocardiogram confirmed atrial fibrillation and pulmonary edema was evident on chest X-ray. The patient was admitted to the medical ward for rate control and diuresis. Heart rate was controlled with metoprolol. An echocardiogram showed evidence of left atrial enlargement without evidence of systolic dysfunction (ejection fraction 60% to 70%). Although the patient's dyspnea and palpitations had resolved and she expressed a desire to return home, the treating team felt that it would be prudent to determine the etiology of her anemia and thrombocytopenia prior to discharge. The evolution of the complete blood count over the course of the admission is summarized in Table 1.

**Table 1:** Summary of the complete blood count during admission

	30 June	1 July	2 July	4 July	6 July	7 July	8 July
Hemoglobin (g/l)	108	106	110	108	124	112	119
White blood cell count (× 10^9^/liter)	2.7	2.5	3.4	2.8	3.0	2.8	2.8
Platelets (× 10^9^/liter)	68	69	82	82	105	82	96

On peripheral smear, there were no blasts, atypical cells or schizocytes. Review of the bone marrow biopsy confirmed the previous findings and ruled out any infiltrative or dysplastic process in the bone marrow. Iron studies were not consistent with either iron-deficiency anemia or with anemia of chronic disease (iron 23 μmol/l; total iron binding capacity 68 μmol/l; ferritin 75.4 μg/l) and reticulocytes were within normal limits (76 × 10^9^/liter). There was no evidence for hemolysis (lactic dehydrogenase 162 U/liter, billirubin total 15.2 μmol/l; billirubin direct 8 μmol/l). B12 (181 pmol/l) and folate (16.6 nmol/l) levels were within normal limits. A careful review of the patient's history did not reveal any systemic causes that might explain the pancytopenia. The patient denied any recent fever or infection. She was also persistently afebrile during the admission. There was no history of recent exposure to toxins or medications associated with marrow failure. A normal urinalysis and a negative sucrose lysis test ruled out the possibility of paroxysmal nocturnal hemoglobinuria.

There was no evidence of enlargement of the spleen or chronic stigmata of liver disease on physical examination. Chart review, however, indicated that an abdominal ultrasound performed 4 months previously had shown mild enlargement of the spleen (splenic diameter of 13 cm) but also some mild cirrhotic changes. However, liver function tests were normal, with the exception of a mildly elevated aspartate aminotransferase (AST) (alanine transaminase 33 IU/liter; AST 48 IU/liter; alkaline phosphatase 65 IU/liter; gamma-glutamyl transpeptidase 21 IU/liter), as was the coagulation profile, international normalized ratio 1.33. Nonetheless, in view of the previous ultrasound findings and the patient having immigrated from Ethiopia, viral hepatitis serologies were ordered and the ultrasound repeated.

The repeat ultrasound demonstrated not only the mild cirrhotic changes but also a solitary hepatic mass. A magnetic resonance imaging scan confirmed a solitary solid mass in region IV of a mildly to moderately cirrhotic liver (Figure 1). Hepatitis serology came back positive for hepatitis C and the α-fetoprotein level was elevated at 30.1 μg/l. Based on these findings, a diagnosis of hepatocellular carcinoma was made. We believe that the mild pancytopenia that the patient exhibited was likely attributable to hepatitis C infection.

**Figure 1:** **Magnetic resonance imaging scan of the abdomen with a hepatocellular carcinoma indicated by the arrow**.

## Conclusion

Previously reported cases of acquired pancytopenia associated with viral hepatitis have occurred in the context of acute hepatitis rather than chronic infection, with bone marrow biopsy usually revealing a markedly hypocellular marrow [1-3]. Given the normocellular bone marrow biopsy result in our patient, it is possible that her pancytopenia resulted from a combination of the T-cell-mediated immune reaction, that is believed to occur with hepatitis virus infection [2,3], and peripheral sequestration from hypersplenism secondary to portal hypertension induced by the cirrhosis. Although, the patient lacked any of the stigmata of portal hypertension on physical examination, the enlargement of the spleen appreciated on ultrasound is likely attributable to this fact.

The pancytopenia work-up performed in the hospital undoubtedly prolonged the duration of the patient's hospitalization. Diuresis, rate control and anticoagulation resolved the symptoms related to atrial fibrillation. However, in view of the fact that outpatient evaluation had failed to identify the etiology of her pancytopenia over a 24-week period, it was felt that a more concentrated effort on an in-patient service would be advisable. We believe that this led to a more rapid diagnosis of hepatocellular carcinoma than would have occurred in the outpatient setting, thus increasing the likelihood of a curative intervention.

## Competing interests

The authors declare that they have no competing interests.

## Authors' contributions

CL and KD contributed equally to the drafting of the text of this case report. Both authors have read and approved the final manuscript.

## Consent

Written informed consent was obtained from the patient for publication of this case report and any accompanying images. A copy of the written consent is available for review by the Editor-in-Chief of this journal.
